# Induction of Resistance of Antagonistic Bacterium Burkholderia contaminans to Postharvest Botrytis cinerea in Rosa vinifera

This article has been retracted.

**DOI:** 10.1155/2022/7134161

**Published:** 2022-06-29

**Authors:** Fengying Shen, Zigang Liu, Chenyang Du, Junhai Yuan, Weigang Wu, Dong Wei

**Affiliations:** ^1^Hebei Key Laboratory of Quality & Safety Analysis-Testing for Agro-Products and Food, Hebei North University, Zhangjiakou City, Hebei Province, China 075000; ^2^College of Agriculture and Forestry Science and Technology, North University of Hebei, Zhangjiakou City, Hebei Province, China 075000

## Abstract

In order to study the problem that grapes are vulnerable to microbial infection and decay during storage, a method based on antagonistic Burkholderia contaminans against postharvest Botrytis cinerea of Rosa vinifera was proposed in this paper. The method tested the resistance induction mechanism of Botrytis cinerea after harvest and determined the fruit decay rate treated by antagonistic Burkholderia contaminans. The results showed that the antagonistic bacterium B-1 had bacteriostatic effect on many common pathogens of fruits and vegetables to a certain extent, and the bacteriostatic range was wide. Among them, the inhibition rate of Fusarium moniliforme was 75.5% and that of Botrytis cinerea was 51.2%. After testing, it can be found that antagonistic bacteria have an inhibitory effect on pathogenic fungi and have an effect on phenylpropane metabolic pathway, reactive oxygen species metabolic pathway, and the activities of other resistance-related enzymes. Through comparison, it can be found that the antagonistic Burkholderia contaminans has a strong antibacterial mechanism against Botrytis cinerea of rose grape after harvest. The fruit treated with antagonistic B Burkholderia B-1 has significantly reduced the decay rate and increased the activity of antibacterial active protein.

## 1. Introduction

Rose grape is famous for its good taste, but it is not easy to keep fresh and easy to rot during storage. Botrytis cinerea is a common disease type after harvest. Due to the low-temperature resistance of the pathogen Botrytis cinerea in the Han Dynasty, it is easy to parasitize on grapes and affect the storage quality of grape (Figure 1). In order to better ensure the quality of grape products, there are anticorrosion technologies in biological control technology, which can improve the resistance to pathogens. The fruit postharvest resistance elicitor can effectively resist pathogens and reduce the degree of decay by stimulating plant disease resistance [1]. In this paper, the antagonistic Burkholderia contaminans was used as the biocontrol strain to study its induction mechanism of postharvest disease resistance of grapes, so as to provide reference basis for the development of postharvest biological control technology of grapes [2].

## 2. Grape Industry and Preservation Technology

Fruits and vegetables account for an important proportion in the diet structure. In recent years, with the improvement of people's quality of life and health awareness, the demand for them has increased accordingly [3]. However, in the postharvest management of fresh fruits and vegetables, due to the lack of perfect preservation technology, the number of decay is huge, resulting in a situation of high yield but no harvest, which not only makes it difficult for fruits and vegetables to realize their due commodity and economic value, but also makes operators lose confidence in this industry. It is reported that the annual loss of fruits and vegetables in China due to improper postharvest management is more than 25% [4]. Because of its soft and juicy characteristics, grapes are more perishable and have greater economic losses in the process of postharvest transportation and storage. Among them, rose grape contains a large number of active substances, so it is very vulnerable to microbial infection in the process of postharvest preservation, which is difficult to maintain until sale, affecting the interests of fruit farmers [5].

At present, there are many kinds of grape storage and preservation technologies studied at home and abroad, mainly divided into physical and chemical methods. Although various technical principles focus on different aspects, they all achieve the purpose of preservation by controlling the process of fruit senescence, controlling the growth and reproduction of pathogenic microorganisms, and controlling internal water loss [6]. At present, the commonly used fresh-keeping methods include SO_2_ and H_2_O_2_ fumigation storage, low-temperature storage, controlled atmosphere storage, and radiation storage. In addition, in recent years, the study of coating a layer of film on the surface of grapes to delay fruit shrinkage and maturity and aging also showed a good fresh-keeping effect. It was found that coating chitosan on the surface of grapes can improve the storage quality of grapes to a certain extent. However, the most common and effective preservation technology in practical production and application is low temperature combined with SO_2_ fumigation [7].

### 2.1. Biological Control of Antagonistic Bacteria against Postharvest Diseases of Grapes

Biological control of pathogenic bacteria is a new research direction rising in recent years. It mainly refers to using the antagonism between microorganisms to select microorganisms that do not harm the host to inhibit the growth of pathogenic microorganisms and control the occurrence of host diseases [8]. The inhibition mechanism of antagonistic bacteria plays an important role in the application of fruits and vegetables. Due to the relatively complex mechanism of antagonistic bacteria, it will interact with pathogens and hosts under the influence of external environmental conditions [9]. The antagonistic effects are produced by the joint action of many factors. In the long-term coexistence of plants and their pathogens, pathogens produce different types of pathogenicity, and plants also form different forms of disease resistance. The production of plant disease resistance can hinder the infection of pathogens to a certain extent, so as to control the occurrence of diseases. There are many factors that can induce plant resistance. As a biological inducer, antagonistic bacteria can induce the resistance of fruits and vegetables to pathogens during postharvest storage, so as to reduce decay [10]. In general, antagonistic bacteria can change the resistance of fruits and vegetables by inducing the activity of resistance-related enzymes, regulating the metabolism of reactive oxygen species, promoting plants to produce defensins, and changing cell structure. It was found that the inoculation of Candida albicans on grape peel could induce the production of phytoalexin [11]. When antagonistic bacteria were used to treat fruits and vegetables, different treatment solutions had different inhibitory effects on pathogens. Fermentation of different antagonistic treatment solutions can have an excellent inhibitory effect on mycosis. When using this method to treat fruits, the control effect will also be improved with the increase of antagonistic concentration in a certain range.

At present, the sterilization technology of fresh-keeping vegetables and fruits abroad mainly adopts the chemical method of low temperature. However, it will increase the drug resistance of pathogenic microorganisms, lead to the accumulation of toxic substances in the human body, and cause environmental pollution. Therefore, it is necessary to develop more practical preservatives to ensure the freshness of fruits and vegetables [12]. In this paper, Burkholderia contaminans of Burkholderia was used as the biocontrol strain to explore the antagonistic mechanism of antagonistic bacteria against postharvest gray mold of grape fruit, so as to lay a foundation for improving the economic value of food use.

### 2.2. In Vitro Inhibitory Effect of Burkholderia on Pathogenic Bacteria of Rosa rugosa

During the postharvest storage of grapes, the rot and deterioration of grapes were caused by fungal infection. The existing preservation technology is to inhibit the growth of pathogenic bacteria, in which Botrytis cinerea is a common pathogen type in postharvest storage of grapes [13]. Because of its low-temperature resistance, it is difficult to treat it by fresh-keeping technology. With the continuous development of microbial control technology, the antagonistic growth curve is explored according to the inhibition effect and principle of postharvest pathogenic bacteria of winter jujube, and the inhibition effect of culture medium on spore is tested based on its different state and time.

#### 2.2.1. Materials, Equipment, and Methods

*(1) Antagonistic Bacteria and Pathogens*. The antagonistic bacteria selected in this experiment is Burkholderia contaminans B-1, which was isolated from the surface of fruits and vegetables through experiments. It was identified by comparing the nuclear dry acid sequences of ribosomal 26SD_1_/D_2_ region and its region and stored at 80°C.

The pathogen is B. cinerea on fresh grapes, which was isolated from naturally occurring fruits and identified by its region [14].

*(2) Reagents and Instruments*. The bacterial culture medium is LB medium: peptone 10.0 g, sodium chloride 5.0 g, yeast extract 10.0 g, and distilled water 1000 ml. The fungal culture medium is PDA medium: potato 200   g, glucose 20 g, agar 15 g, and distilled water 1000 ml.

Ls-b50l-i vertical pressure steam sterilizer; Dhp-9272 electric constant temperature incubator (Shanghai Yiheng Technology Co., Ltd.); Bsd-wf2200 oscillation incubator (Shanghai Boshun Industrial Co., Ltd.); Gl-20   (g-1i centrifuge of Shanghai Anting Scientific Instrument Factory); Jeoljem6490lv scanning electron microscope (Nippon Electronics Co., Ltd.) [15].

*(3) Method*. The antagonistic bacteria were activated on LB solid medium, and the activated antagonistic single bacteria were selected and cultured at 28°C and 200 R/min according to 1% of the inoculation amount. The concentration of bacterial solution was tested at different time points, and the regression equation of *Y* = *aX* + *b* was obtained by SAS 9.0 according to the light absorption value and concentration to determine the growth curve of antagonistic bacteria [16]. This process was repeated for three times. The effect of antagonistic bacteria on the antibacterial ability of sporangium in different time periods needs to be inoculated into the culture medium, respectively, and the experimental results should be observed according to the time of 24 h, 48 h, 72 h, 96 h, and 120 h. The effect of antagonistic bacteria on the bacteriostasis of sporangium existed in different time periods. After the antagonistic bacteria were cultured for 24 hours, the antagonistic culture medium, the bacterial suspension, the filter solution, and the heat killing solution were used, respectively. Treatment method: Dip 20  *μ*L of treatment solution on the PDA plate. After drying, inoculate the spore mycelium block with a diameter of 5 mm in the center of the plate, and culture it at a constant temperature of 26°C for 5-7 d. Wait until the mycelium grows to the edge of the culture dish for inspection, and repeat the experiment three times. The antibacterial effect of antagonistic bacteria is different under different temperature conditions. It is necessary to take the antagonistic culture medium cultured in a shaking flask at 28°C for 24 hours under the conditions of 37°C, 45°C, 50°C, 80°C, and 100°C for 30 minutes, and then, use the Oxford cup method to measure the diameter of the antibacterial circle under different conditions (the method has the same effect as the antibacterial ability). Each treatment is repeated for 3 times, and the experiment is repeated for 3 times. The antagonistic culture medium cultured in shaking flask at 28°C for 24 hours was adjusted to pH 1, 4, 7, 9, and 14, respectively, and then stood for 24 hours [17]. The diameter of antagonistic circle under different conditions was measured by Oxford cup method, and the test was repeated three times. The hyphae of common pathogens of fruits and vegetables with a diameter of 5 mm were inoculated at 3.5 cm from the edge of the Petri dish on the PDA plate. Pick the activated single bacterial colony with the inoculation ring, and draw a line 3.5 cm away from the pathogen (the control is not drawn). All treatments were cultured in the dark in a 26°C incubator. After 6 days, the radius length of pathogenic bacteria colonies growing on the scribed side was measured, and the inhibition rate was calculated. Three repetitions were set for each treatment, and the experiment was repeated three times.

### 2.3. Results and Analysis

Use Excel 2007 and SAS 9.0 to statistically analyze the data, calculate the standard and draw the drawing, and analyze the significance of the data. *P* < 0.05 indicates that the difference is significant.

#### 2.3.1. Determination of Antagonistic Growth Curve

According to the concentration measured by dilution plate method and its corresponding 0D_600_ value, the regression equation of 1G live bacteria number of antagonistic B-1 is determined as *Y* = 2.6911*X* + 7.7307, and *R*^2^ value is 0.8978. The growth curve of antagonistic bacteria with inoculation time is shown in Figure 2. Within 8 h after inoculation, antagonistic bacteria grow slowly, and enter rapid growth after 8 h to 24 h: long state, logarithmic growth period, slow growth after 24 h, and enter stable period. At 48 h after inoculation, the concentration of the bacteria reaches the maximum value of 1.003 × 10^13^cfu/mL, and enters decay period after 72 h. With the extension of culture time, the number of viable bacteria decreases gradually [18].

#### 2.3.2. Effect of Antagonistic Culture Medium at Different Time on Antibacterial Ability of Spores

The results showed that compared with the control, the culture medium with culture time of 24 h, 48 h, 72 h, and 96 h could inhibit the growth of B. cinerea in varying degrees. However, the size of the bacteriostatic circle produced by the culture medium at different times is different. The bacteriostatic circle of the culture medium is the clearest at 24 h, and its diameter is the largest (Table 1), which is 2.81 cm, followed by 48 h. With the extension of the culture time, the bacteriostatic circle gradually becomes blurred and narrowed. At 120 h, the bacteriostatic circle becomes very blurred, and the bacteriostatic effect is not obvious [19].

#### 2.3.3. Antibacterial Ability of Different Antagonistic Treatment Solutions to Botrytis cinerea

It was found that the culture medium and bacterial suspension could completely inhibit the growth of Botrytis cinerea after 5 days of culture. Botrytis cinerea treated with filter solution, heat killing solution, and LB medium grew to the edge of the culture dish, which was no different from the control [20].

When the bacteriostatic circle diameter was slightly higher than that of the control when the bacteriostatic circle diameter was higher than that of the control when the bacteriostatic circle diameter was higher than 50°C (Figure 3), the bacteriostatic circle diameter was slightly lower than that of the control when the bacteriostatic circle diameter was higher than that of the control when the bacteriostatic circle temperature was higher than 50°C.

The bacteriostatic effect of antagonistic bacteria under different pH conditions is shown in Figure 4. It can be seen that the bacteriostatic circle diameter of antagonistic bacteria under neutral conditions (pH =7) is the largest, which is 2.9 cm, and the bacteriostatic effect under acidic conditions is reduced. When pH is 1, the diameter is 2.0 cm, and alkaline conditions have a significant impact on the bacteriostatic effect of antagonistic bacteria [21]. When pH is 9, the diameter is 1.7 cm, and when pH reaches 14, there is no bacteriostatic circle, and the bacteriostatic effect is lost.

As shown in Figure 5, antagonistic bacteria have a certain inhibitory effect on fruit and vegetable pathogens. The inhibition effect on *Fusarium moniliforme* was the best, and the inhibition rate was 75.5%. Compared with other pathogens, antagonistic bacteria have a medium to upper level in the inhibition effect of pathogen *B. cinerea* in this experiment, and the inhibition rate can reach 51.2%.

Botrytis cinerea is a common disease in grape postharvest storage. The pathogen parasitized on the fruit and led to grape decay. Through the study of antagonistic bacteria B. contaminans and B. cinerea, a series of experiments showed good antibacterial effect. During the experiment, both temperature and pH value had an impact on the antibacterial activity of antagonistic bacteria, and the antagonistic bacteria had a good antibacterial effect between the lethal temperature, indicating that the bacteria was acid resistant. The final experiment verified the effect of antagonistic bacteria on pathogenic bacteria, which can play a good antibacterial effect, and the antibacterial rate reached 51.2%. It is speculated that the bacteria has a certain potential in the storage and preservation of fruits and vegetables [22].

## 3. Inhibitory Effect of Antagonistic Bacteria on Postharvest B. cinerea of Rosa vinifera

Due to the thin skin and high juice content of rose grape, it is difficult to store it. And the preservation technology is closely related to pathogens. It is necessary to start with antagonistic bacteria to reduce the amount of bacteria before grape storage, so as to improve the preservation effect of fruits and vegetables after storage. The fixed value state of antagonists and pathogens in fruit wound was observed, and the related indexes were evaluated.

### 3.1. Materials, Strains, and Reagents

Rosemary grapes are collected from rosemary planting base in Taigu County, Shanxi Province. They are picked when they reach the commercial maturity. On the day of picking, they are transported back to the laboratory for pre cooling and stored in 0°C cold storage. Holderia was isolated from the surface of apricot fruit by our laboratory and was identified according to the nucleotide sequence alignment and physiological and biochemical characteristics of ribosomal 26S D1/D2 region and its region; Botrytis cinerea was isolated from naturally occurring grape fruits and was identified by its region and morphological characteristics. The bacterial culture medium is LB medium: yeast extract 10.0 g/l, peptone 10.0 g/l, and sodium chloride 5.0 g/L. The fungal culture medium is PDA medium: potato 200 g/l, glucose 20 g/l, and agar 15 g/L. P-Aminobenzene Sulfonic Acid, 3,5-Dinitrosalicylic acid, potassium sodium tartrate, catechol (Tianjin Guangfu Fine Chemical Research Institute); Guaiacol *α*- Naphthylamine, kelp protein, chitin, riboflavin, snail enzyme (Beijing solabao Technology Co., Ltd.) [23].

### 3.2. Method

#### 3.2.1. Preparation of Fermentation Stock Solution

After the antagonistic bacterium B-1 stored at -80°C was activated in LB solid medium, a single colony of antagonistic bacterium B. contaminans B-1 on the activated LB solid medium was selected and cultured in 300/1000 mL LB liquid medium at 200 r/min for 24 hours.

#### 3.2.2. Preparation of Mold Spore Suspension

After Botrytis cinerea was cultured on PDA plate for 7 days, the conidia were scraped, and the spore suspension with the concentration of 1.0 × l0^5^spores/mL was prepared with sterile water by blood cell counting method.

The calculation formula is *N* = ∑*C*/nn_1_ + 0.1n_2_nd; during application, it is necessary to ensure that the diluent is within the appropriate range, which is calculated according to the following formula: *N* = ∑*C*/[n1 + n0.1∗n2n]∗ndn.

Calculate the required solution dilution ratio according to the dilution:

(1) $$\begin{array}{c} N=\sum C/\text{n}{\text{n}}_{1}+0.1{\text{n}}_{2}\text{nd}=\frac{232+244+33+35}{\left[2+\text{n}0.1*2\text{n}\right]*10^{-2}}=\frac{544}{2.2*10^{-2}}. \end{array}$$

#### 3.2.3. Sample Treatment of Fruit Storage Effect

Select the Rosa vinifera with the same maturity and no mechanical damage in appearance, soak it in the culture solution of antagonistic LB with different concentrations ((a) fermentation stock solution; (b) diluted 5 times fermentation solution; and (c) diluted 10 times fermentation solution) for 2 min (the control is not treated), place it in the sterilized plastic basket (20 strings per basket, about 20 fruits per string), store it under the condition of 0°C for 70 days, and then check it. The experiment was repeated three times.

#### 3.2.4. Determination of Indicators of Substances Related to Fruit Resistance and Sample Treatment

About 750 Rosa vinifera grapes without mechanical injury and with the same maturity were selected and randomly divided into control group and treatment group. The fruits of the two groups were soaked in 2% sodium hypochlorite solution for 2 minutes, dried with sterile air, and stabbed a wound with a diameter of 4 mm and a depth of 3 mm at the equator with a sterilization needle, one wound for each grape. In the treatment group, 30 *μ*L of 24-h fermentation broth of contaminans was added to the wound, and in the control group, 30 *μ*L of sterile water was added. After 2 hours, add 15 *μ*L mold spore suspension at each wound, dry it with sterile air, and then incubate it in a 25°C incubator for 6 days. 50 fruits of the treatment group and the control group were taken every day. The pulp at the junction of the wound lesion and the healthy tissue were used as the experimental material. After liquid nitrogen treatment, it was stored at -80°C for use. The experiment was repeated three times [24].

### 3.3. Determination of Fruit Storage Effect

The rotten degree of fruit and stem after 70 days storage was investigated. The fruit was graded according to the rotten degree and weighed. The rotten rate of stem and rotten index of fruit were calculated according to (1) and (2). The fruit stalk is mildewed to rot, and it is normal without mildewing.

(2) $$\begin{array}{c} \text{Fruit rot rate}/\%=\frac{\text{Rotten fruit count}}{\text{Total number of fruit stems}}*100\text{ n}1\text{n}. \end{array}$$

According to the degree of fruit decay, it is divided into 5 grades, and the grading standards are as follows: grade 0, the fruit is intact without any decay; grade 1, there are slight spots on the fruit surface, and the rotten area accounts for less than 1/3 of the fruit surface; grade 2, the fruit surface has obvious decay, and the decay area accounts for about 1/3 ~ 1/2 of the fruit surface; grade 3, the fruit rots more than 1/2 of the fruit surface, but the fruit still has a certain hardness; and grade 4, the whole fruit is completely rotten. After grading the fruit, weigh the quality, respectively.

(3) $$\begin{array}{c} \text{Pulp rot index}/\%=\frac{\sum \text{n}\text{Proportion of rotten fruits at all levels}*\text{The representative value of this classn}}{1*\text{Representative value at all levels}}*100\;\text{n}2\text{n}. \end{array}$$

## 4. Result Analysis

### 4.1. Inhibitory Effect of Antagonistic Bacteria on Natural Decay of Rose Grape during Postharvest Storage

Antagonistic bacteria could inhibit the natural decay of rose after harvest. It can be seen from Figure 6 that after Rosa vinifera was treated with antagonistic fermentation broth and stored at 0°C for 70 days, three different concentrations of fermentation broth can effectively inhibit grape decay (*P* < 0.05). Most of the stem and pulp of the control fruit were mildewed and rotted, while the degree of decay was significantly reduced after the treatment with antagonistic bacteria (Burkholderia contaminans). Among them, the storage effect of 5 times diluted fermentation broth is the best, followed by the effect of fermentation stock broth, and the effect of 10 times diluted fermentation broth is relatively poor. The decay rate of the control stem was 100%, and the decay index of the pulp was 67.14%. However, when the fermentation broth was diluted five times, the fruit stem decay rate was only 30.42%, the pulp decay index was only 3.21%, the fruit stem decay rate was reduced by 69.58%, and the pulp decay index was reduced by 63.93%.

### 4.2. Effects of Antagonistic Treatment on PAL, , and PPO Activities of Grape Fruit

As the key enzyme in the first step of phenylpropanoid metabolism, PAL is involved in the biosynthesis of disease resistance-related substances such as plant lignin, phytoalexin, and phenols. The highly toxic quinones produced by PPO oxidizing phenols can limit and kill invading pathogenic microorganisms. POD is closely related to the synthesis of lignin and phytoalexin in plants, and the removal of H_2_O and $O\bar{2}•$ is harmful to plant cells.

It can be seen from Figures 7, 8, and 9 that the PAL activity of the control and treatment reached the peak on the first day and there was a similar peak. In the following 1 ~ 5 days, the PAL activity of the fruits treated with antagonistic bacteria was stable higher than that of the control, and the difference between the two narrowed 5 days after treatment. The activity of the treatment group and the control group showed an upward trend as a whole. There was little difference in the enzyme activity in the first three days. From the third day, the POD activity of the treatment group increased rapidly, and the value was significantly higher than that of the control. By the fifth day, the difference between the two groups decreased. During the whole storage period, the PPO activity of the treated group was significantly higher than that of the control. Compared with the control, the PPO activity of the experimental group began to rise rapidly on the first day, reached the peak on the third day, and then began to decline.

### 4.3. Control Effect of Antagonistic Bacteria on Natural Decay of Grapes after Harvest

Grape fruits were treated and stored with different chemical treatment solutions. The results are shown in Table 2. Under different temperature conditions, different treatment solutions can inhibit grape fruit to a certain extent, and the nutrient solution diluted by 5 times has the best storage effect. And under different temperature conditions and storage for different days, compared with the control fruit stem, the decay rate decreased the antagonistic bacteria. The anticorrosion effect of suspension was only 5 times higher than that of culture.

### 4.4. Discussion

Some studies have found that some antibacterial strains can produce bacteriostatic circles in vitro, but they have no bacteriostatic effect when applied to fruits. The main reasons are as follows: some bacteria can only produce bacteriostatic substances in vitro, but not in vivo; the complex and changeable environment of living wound is not suitable for some bacteria to survive or weaken their vitality, including the antieffect. In the experiment, compared with the control group, the SOD activity of antagonistic grape fruit increased rapidly on the first day of storage, while the cat activity decreased significantly, which promoted the accumulation of H_2_O_2_ in grape fruit cells. The rapid accumulation of H_2_O_2_ plays an important role in the disease resistance response of plants. It not only has the direct function of antiviral microorganisms, but also its existence can cause damage to pathogens. In the later stage of storage, the cat activity of the treatment group was significantly higher than that of the control group, which eliminated the excessive H_2_O_2_ accumulated in the pulp, so as to avoid the body damage caused by excessive reactive oxygen species in the fruit. In conclusion, as a biological control technology, Burkholderia contaminans B-1 treatment can significantly improve the disease resistance of grapes in postharvest storage and achieve the purpose of anticorrosion and fresh-keeping.

According to the above experiments, antagonistic bacteria, as a biological bactericide, have a good inhibitory effect on staphylococcal mycosis. However, because it is a living bacterial agent, it wants to promote the industrialized production of the device. A large number of cultures are needed to screen the best medium formula for the basic nutrients needed by antagonists, so as to provide a more perfect theory for the preservation of fruits and vegetables.

The antagonistic bacteria were inoculated into 100/250 mL liquid medium after being activated in LB solid medium and cultured in shaking flask at 28°C 200/min for 24 h to prepare seed solution. The addition amount of various carbon sources to be tested is 1%, and 1I% YNB is the basic nitrogen source. Inoculate 1% of the inoculated amount into a 50/250 mL triangular flask, incubate for 24 hours under the condition of 200/min at 28°C, measure the value of 0D_600_ with a spectrophotometer, and repeat each treatment for 3 times.

#### 4.4.1. Screening of the Best Nitrogen Source

Add 1% of all tested nitrogen sources, and take the selected best carbon source as the carbon source. Each treatment was repeated 3 times.

The composition of antagonistic medium was optimized by secondary general rotation combination. The test factors include carbon source, nitrogen source, and other components, and each factor contains five levels. The OD_600_ value of antagonistic growth dilution 10 times was used as the response design (see Table 3 for the specific code), and each treatment was repeated three times.

The test data were counted by Design-Expert 8.0.6 statistical software and processed in group mode. The OD_600_ value was measured after 10 times dilution.

As shown in Table 4, among the utilization capacity of antagonists to different carbon and nitrogen sources, it can be seen that the utilization capacity of antagonists to malt leaching powder is the highest, which is significantly higher than that of other carbon sources. The utilization ability of yeast extract in nitrogen source was the strongest, which was significantly higher than that of other nitrogen sources.

According to Table 5, the concentration of carbon source sucrose is between 2.0 and 3.0%, and the antagonistic culture density is the largest. When the concentration of nitrogen source was 4.0%, the culture density was the highest.

The best level of each factor is determined by using Design-Expert 8.0.6 statistical software. According to the regression equation:

(4) $$\begin{array}{c} \begin{array}{c} Y=1.35+0.099\;X_{1}+0.12\;X_{2}-0.013\;X_{3}-0.002486\;X_{4}-0.12\;\\ X_{1}X_{2}+0.013X_{1}X_{3}+0.004729X_{1}X_{4}+0.022X_{2}X_{3}-0.002687\\ X_{2}X_{4}+0.019X_{3}X_{4}-0.14X_{1}^{2}-0.1X_{2}^{2}-0.075X_{3}^{2}-0.098X_{4}^{2} \end{array} \end{array}$$

Verify the regression coefficients. It is *X*1 = 0.115, *X*2 = 0.538, *X*3 = −0.002, and *X*4 = −0.018. The level before transformation into coding is as follows: malt extract powder is 2.11%, yeast extract is 1.9%, and the corresponding*y*value is 1.38901. In order to verify the culture conditions, 2.11% malt powder and 1.9% yeast extract were used to dilute the obtained bacterial solution, and the OD600 was 1.31. The error is 5.0%, indicating that the culture method is feasible.

## 5. Conclusion

In conclusion, when the antagonistic bacteria Burkholderia contaminans B-1 and Botrytis cinerea confront in vitro, the bacteriostatic circle diameter of 24-h culture medium and culture stock solution is the largest and clearest, and the inhibitory effect will be shown only when they are in certain contact with the pathogen; that is, on the one hand, the bacteriostatic mechanism of this bacterium is to produce bacteriostatic substances. UV irradiation, high-temperature treatment, and adjusting the pH of culture medium can all have a certain impact on the antibacterial activity of antagonistic bacteria, but it will lose its antibacterial effect only in extreme environment, that is, high temperature and high alkali, while the normal living environment has little impact on its antibacterial activity. When Botrytis cinerea spores were treated with antagonistic bacteria, the spore germination and the secondary length of bud tube were significantly inhibited, and the degree of inhibition increased with the increase of antagonistic concentration. Under scanning electron microscope, it was also found that Botrytis cinerea mycelium was seriously shrunk and deformed compared with the control. In addition, antagonistic B-1 has antibacterial effect on a variety of common pathogens in fruits and vegetables to a certain extent, with a wide range of inhibition, in which the inhibition rate of Fusarium moniliforme can reach 75.5%, and that of Botrytis cinerea is 51.2%. Antibacterial B-1 treatment increased the activities of resistance-related enzymes PPO, POD, PAL, CHI, GIU, and SOD in grape fruit to a certain extent, delayed the peak time of cat enzyme activity, and increased the accumulation of active H_2_O_2_. The changes of these resistance-related active substances enhanced the resistance of fruit to pathogens. The optimal formula of antagonistic growth was obtained by response surface test, namely, 2.11% malt extract and 1.9% yeast extract.

Although the effect of bile storage of postharvest rose grape with antagonistic bacteria is worse than that of commonly used chemical agents, and the strains used in this experiment are currently limited to laboratory research, they have shown their unique advantages. Firstly, compared with chemical agents, biological agents have the advantages of no pollution to the environment, no resistance, and no damage to human health and have great application potential. Although the research on antagonistic bacteria B. contaminans in this experiment is in the early stage, all exploration and research will be devoted to its practical application in grape storage and preservation.

## Figures and Tables

**Figure 1:** Antimicrobial guide.

**Figure 2:** Growth dynamics of antagonists in LB medium.

**Figure 3:** Effect of temperature on antagonistic inhibition zone.

**Figure 4:** Effect of pH on antagonistic circle.

**Figure 5:** Antagonistic ability of B. cinerea against various pathogens.

**Figure 6:** Inhibitory effect of antagonistic bacteria on postharvest storage decay of grapes.

**Figure 7:** Effect of antagonistic treatment on pal activities of postharvest grapes.

**Figure 8:** Effect of antagonistic treatment on POD activities of postharvest grapes.

**Figure 9:** Effect of antagonistic treatment on PPO activities of postharvest grapes.

**Table 1:** Effects of different culture time on bacteriostatic circle of spores.

Incubation time (h)	Bacteriostatic circle diameter (cm)
24	2.81 ± 0.34a
48	2.26 ± 0.33b
72	2.06 ± 0.28c
96	1.79 ± 0.37d
120	1.62 ± 0.21e

Note: the significance test is conducted at the level of 0.05, the same below.

**Table 2:** Control effects of different treatment solutions of B. contaminans on grape stem and pulp.

Treatment	Control effect	
	Fruit stalk(%)	Flesh(%)
	26°C 16°C 0°C	26°C 16°C 0°C
Culture stock solution	28.96c 33.07d 76.47b	41.29c 26.97e 58.75c
Dilute 5 times	61.80a 57.37b 83.33a	59.60b 67.15b 5.22a
Dilute 10 times	25.00d 43.75c 64.29d	37.22d 48.21d 70.23b
Bacterial suspension	61.23a 71.56a 82.34a	70.02a 73.24a 89.31a
Supernatant	45.18b 58.49b 66.17c	37.19d 59.67c 69.48b

**Table 3:** Test factor level and coding table.

Code	Carbon source (%)	Nitrogen source (%)	Inorganic salt 1 (%)	Inorganic salt 2 (%)
-2	0.0	0.0	0.0	0.0
-1	1	0.75	0.0025	0.0025
0	2	1.5	0.05	0.05
1	3	2.2	0.0075	0.0075
2	4	3.0	0.10	0.1
△j	1	0.7	0.0025	0.0025

**Table 4:** Utilization capacity of antagonists to carbon and nitrogen sources.

Carbon source	OD_600_	Duncan's test^a^	Nitrogen source	OD_600_	Duncan's test^a^
Lactose	0.106	d	Fish peptone	0.278	h
Sucrose	0.522	bc	Soybean peptone	2.337	ab
Malt dust	0.447	d	Polypeptone	2.265	b
Glucose	0.429	bc	Yeast extract	2.385	a
Malt extract	1.454	a	Urea	0.568	g
Contrast	0.0417	d	Contrast	1.415	e

**Table 5:** Effects of different carbon and nitrogen sources on antagonistic culture density.

Concentration(%)	Nutrients			
	Malt extract		Yeast extract	
	OD_600_	Duncan's test^a^	OD_600_	Duncan's test^a^
0	2.185	ab	1.443	e
0.5	2.278	ab	2.187	d
1.0	2.276	ab	2.331	c
1.5	2.347	ab	2.519	b
2.0	2.355	ab	2.661	a
2.5	2.345	ab	2.694	a
3.0	2.470	a	2.689	a
3.5	2.002	b	2.707	a
4.0	1.175	c	2.716	a

## Data Availability

The labeled data set used to support the findings of this study is available from the corresponding author upon request.
